The article "Pixel-Wise Classification in Hippocampus Histological Images" was published in 2021. Journal: Comput Math Methods Med.

# Pixel-Wise Classification in Hippocampus Histological Images

**DOI:** 10.1155/2021/6663977

**Published:** 2021-05-20

**Authors:** Alfonso Vizcaíno, Hermilo Sánchez-Cruz, Humberto Sossa, J. Luis Quintanar

**Affiliations:** ^1^Departamento de Ciencias de la Computación, Universidad Autónoma de Aguascalientes, Aguascalientes 20131, Mexico; ^2^Centro de Investigación en Computación, Instituto Politécnico Nacional, Ciudad de México, Mexico; ^3^Departamento de Fisiología y Farmacología, Universidad Autónoma de Aguascalientes, Aguascalientes 20131, Mexico

## Abstract

This paper presents a method for pixel-wise classification applied for the first time on hippocampus histological images. The goal is achieved by representing pixels in a 14-D vector, composed of grey-level information and moment invariants. Then, several popular machine learning models are used to categorize them, and multiple metrics are computed to evaluate the performance of the different models. The multilayer perceptron, random forest, support vector machine, and radial basis function networks were compared, achieving the multilayer perceptron model the highest result on accuracy metric, AUC, and *F*_1_ score with highly satisfactory results for substituting a manual classification task, due to an expert opinion in the hippocampus histological images.

## 1. Introduction

The study of the hippocampus region has been of particular interest because of its relationship with memory and learning processes [1, 2], its volume as an indicator for Alzheimer's disease [3], personality disorder [4], neurological disorders derived from strokes [5–9], and drug addiction effects [10], to mention a few.

Most common hippocampal quantification techniques are based in MRI images [11, 12] for volumetric calculation and histological images [13, 14] for neural cell counting.

However, determining hippocampal volume in histological images is a challenging labour, on the one hand because image conditions are not always good and hippocampus section is of an irregular shape that is only a few pixels thick, which makes this labour an intensive and time-consuming task that demands the help of an expert to correctly identify the area of interest and so be able to determine hippocampus volume.

On one hand, pixel-wise classification has been used broadly for task such as mitosis detection in histological breast images for cancer detection [15–17], gland segmentation of prostate histology images [18], and nuclei segmentation [19], among others, where the solution range goes from digital image processing approaches used in combination with ML techniques to convolutional neural networks.

On the other hand, studies on hippocampus region have been performed exhaustively using magnetic resonance images from humans and rats, to perform segmentation tasks by applying several methods such as atlas based [20–23], a combination with support vector machines (SVMs) [24], and patch-based approaches [25], among others [26–29].

The article "Pixel-Wise Classification in Hippocampus Histological Images" was published in 2021. Journal: Comput Math Methods Med.

Even though each published work reports improvements over previous approaches on their own image source type and task types, as far as we know with our deep search in the literature, to perform a pixel-wise classification on hippocampus structure from rat brain histological images cuts, using the coronal anatomical plane, has not been done before. Mesejo et al. [30] perform a segmentation endeavour by using deformable models and random forest (RF) from Allen Brain Atlas [31] image repository using the sagittal anatomical plane. Senyukova et al. [32] do atlas-based segmentation on several brain sections with RF and Markov Random Fields on Nissl-stained histological sections of mouse brains. And Riklin-Raviv et al. [33] propose a slice-by-slice segmentation with three-dimensional Gaussian mixtures and level sets where the successful segmentation of one section provides a prior for the subsequent one, assuming that the segmentation of few sparsely sampled slices is done manually.

This work reports the implementation of a computer vision method to extract pixel features and use them along with several machine learning (ML) techniques such as multilayer perceptron network (MLP), SVM, radial basis function network (RBFN), and RF, to perform pixel-wise classification on rat brain histological images using the coronal anatomical plane to correctly identify the hippocampus structure and facilitate its measurement.

## 2. Materials and Methods

The images used in this work are supplied by the Pharmacology Department of the Autonomous University of Aguascalientes. These images are serial coronal sections of approximately 6 *μ* thick, from male rat brains of the Sprague Dawley strain around 8-12 weeks old with a weight of 250-330 g. The cuts are stained with a specific chemical dye, and in this case hematoxylin-eosin is employed, to create contrast on the seeked anatomical structure.

A total of 25 images were digitized from an optical microscope with a magnifying glass of 0.67x, using an LGE LM-X520 camera model that was configured with an ISO speed rating of 100, a focal length of 3.5 mm, and a variable exposure time ranging from 1/60 s to 1/30 s. Each image was captured at 4161 × 3120 pixels and was saved originally in JPEG format.

When performing a visual inspection on these images, several conditions can be identified:

- No relevance on a specific colour for detecting anatomical structures
- Different lighting effects: some images are brighter than others
- Fuzziness of the hippocampus boundaries
- Variability of hippocampus' shape and orientation
- Cutoff of regions and presence of markings such as scraps, tears, and streaks in tissue
- Rotated and uncentred brain position

Examples of some of these characteristics are shown in Figure 1.

The article "Pixel-Wise Classification in Hippocampus Histological Images" was published in 2021. Journal: Comput Math Methods Med.

Our methodology for hippocampus pixel classification consists of four consecutive steps, as depicted in Figure 2. The first step uses image processing to enhance hippocampus region. The second step characterizes each pixel as a 14-dimensional vector. Those vectors constitute the features used by the classification algorithms. After all images have been characterized, the third step begins. At this step, the training, validation, and test set are created. The last step involves feature classification to differentiate between a nonhippocampus pixel and hippocampus pixel. The details of each of these steps are now described.

### 2.1. Image Conditioning and Preprocessing

The provided images contain ample dark areas, since brain image is swiveled and given the large image dimensions, it is necessary to condition them in order to speed up its preprocessing step. Therefore, images are straightened and only brain image is kept along with its aspect ratio. It is determined that an image size average of 1024 × 832 pixels is big enough to preserve hippocampus pixels and small enough to perform a fast preprocessing step. An example of the conditioning phase is displayed in Figure 3. Finally, the coordinates that make up the main hippocampus bounding box are annotated.

Because of the ample differences between hippocampus images and the image conditions explained in previous section, a preprocessing phase is performed in order to enhance hippocampus region and extract meaningful information to construct the features that will be used later in the classification step. This phase is based in the procedure employed in Vega et al. [34] and Marin et al. [35]. However, given the difference between the images and their respective domain field, the procedure has to be tailored to generate suitable images. Next, the details of the preprocessing step are described.

#### 2.1.1. Colour Independence

Histological cuts contain different colours because of the type, amount of dye, and the exposure time given to the tissue. Consequently, pixels differ in colour and intensity despite belonging to the same hippocampus region. For this reason, the input image is converted from an original RGB colour space to a Hue Saturation Value (HSV) colour space, extracting the Value Channel (VC) to better capture the full range of the different colours that belong to the hippocampus and to make it independent from the illumination of the sample images. Then, the image is cropped to the annotated bounding box to be furthered processed. *I*_*V*_ denotes the resultant image for future references. Because of the nature of VC, the hippocampus region is represented by dark colour pixels which correspond to values close to zero. In order to emboss them, image is negated having *I*_NV_ as result.

(1) $$\begin{array}{c} I_{\text{NV}}=255-I_{V}. \end{array}$$

Figures 4(a) and 4(d) show an example of this phase.

The article "Pixel-Wise Classification in Hippocampus Histological Images" was published in 2021. Journal: Comput Math Methods Med.

#### 2.1.2. Background Homogenization

Since the background is not homogeneous, a mean filter followed by a convolution with a Gaussian kernel followed by a histogram correction operation is applied. This phase is performed in the same way that [34] does background homogenization but working with an *I*_NV_ image. The resulting image of this phase is denoted as *I*_*H*_, and an example of the outcome is presented in Figures 4(b) and 4(e).

#### 2.1.3. Hippocampus Enhancement

Hippocampus enhancement is performed by applying a top-hat transformation.

(2) $$\begin{array}{c} I_{\text{HE}}=\gamma \left(I_{H}\right), \end{array}$$

where *γ* is a morphological opening using a disc of eight pixels in radius, thus removing most anatomical structures not belonging to hippocampal region and yielding better results than performing a boundary detection with algorithms like Canny, Prewitt, and Sobel. Figures 4(c) and 4(f) exhibit an example of the procedure applied in this phase.

### 2.2. Feature Extraction

The purpose of this step is to perform a pixel characterization in terms of some quantifiable measurements that can be used latter in the classification step. To accomplish this task, unlike Marin et al. and Vega et al. whom used seven and five functions, respectively, in this work, a total of fourteen functions are used. Our method uses some variants that are described. The first five features are as follows: *f*_1_, *f*_2_, ⋯, *f*_5_, which are based on the pixel's grey-level information available. In this work, we find that the features calculated from *I*_HE_ produce more meaningful representation of hippocampus pixels. The features are outlined as follows: considering a squared pixel region of size *w* × *w* taken from *I*_HE_ and centred at pixel (*x*, *y*), we have the following:

*f*_1_ is the value of the pixel being characterized at position (*x*, *y*) subtracted from the smallest value of the squared region

(3) $$\begin{array}{c} f_{1}\left(x,y\right)=I_{\text{HE}}\left(x,y\right)-\begin{array}{c} \min\\ \left(s,t\right)\in S_{x,y}^{9} \end{array}\left\{I_{\text{HE}}\left(s,t\right)\right\}. \end{array}$$

*f*_2_ is the largest value of the squared region subtracted from the value of the pixel being characterized at position (*x*, *y*)

(4) $$\begin{array}{c} f_{2}\left(x,y\right)=\begin{array}{c} \max\\ \left(s,t\right)\in S_{x,y}^{9} \end{array}\left\{I_{\text{HE}}\left(s,t\right)\right\}-I_{\text{HE}}\left(x,y\right). \end{array}$$

*f*_3_ is the value of the pixel being characterized at position (*x*, *y*) subtracted from the average value of the squared region

(5) $$\begin{array}{c} f_{3}\left(x,y\right)=I_{\text{HE}}\left(x,y\right)-\begin{array}{c} \text{mean}\\ \left(s,t\right)\in S_{x,y}^{9} \end{array}\left\{I_{\text{HE}}\left(s,t\right)\right\}. \end{array}$$

*f*_4_ is the value of standard deviation of the squared pixel region characterized at position (*x*, *y*)

(6) $$\begin{array}{c} f_{4}\left(x,y\right)=\begin{array}{c} \text{stdDev}\\ \left(s,t\right)\in S_{x,y}^{9} \end{array}\left\{{\text{I}}_{\text{HE}}\left(s,t\right)\right\}. \end{array}$$

*f*_5_ is the value of the pixel being characterized at position (*x*, *y*)

(7) $$\begin{array}{c} f_{5}\left(x,y\right)=I_{\text{HE}}\left(x,y\right). \end{array}$$

Then, for the next two features, *f*_6_ and *f*_7_, we use the first two Hu moment invariants [36] denoted by *ϕ*_1_ and *ϕ*_2_. These are computed from *I*_Hu_ image, which is obtained by multiplying a squared pixel region of 17 × 17 size from *I*_HE_ and an equal dimension matrix of Gaussian values, whose mean is 0 and variance is (1.7)^2^; then, *I*_Hu_ is given by

(8) $$\begin{array}{c} I_{\text{Hu}}\left(i,j\right)=I_{\text{HE}}^{S_{x,y}^{17}}\left(i,j\right)\times G_{0,1.7^{2}}^{17}\left(i,j\right). \end{array}$$

With these choices of parameters, the 9 × 9 central values in Gaussian matrix contain 97% of the area of the represented Gaussian distribution, making the remainder values being close to 0. The effect of this multiplication is that the values become sensitive for describing hippocampal and nonhippocampal central pixels. Given that *ϕ*_1_ and *ϕ*_2_ computation can take nonpositive and zero values, *f*_6_ is defined as

(9) $$\begin{array}{c} f_{6}=\left\{\begin{array}{cc} \log\left(\phi_{1}\right), & \text{if}\phi_{1}>0,\\ -\log\left(\left|\phi_{1}\right|\right), & \text{if}\phi_{1}<0,\\ 0, & \text{otherwise}, \end{array}\right. \end{array}$$

and *f*_7_ is defined as

(10) $$\begin{array}{c} f_{7}=\left\{\begin{array}{cc} \log\left(\phi_{2}\right), & \text{if}\phi_{2}>0,\\ -\log\left(\left|\phi_{2}\right|\right), & \text{if}\phi_{2}<0,\\ 0, & \text{otherwise}. \end{array}\right. \end{array}$$

Given that images contain other brain regions of similar shape and that image conditions are extremely variant, a set of extra seven features are used to acquire even more descriptive pixel information that can help better distinguishing between the seeked hippocampus section and the alike structure.  Figure 5 illustrates the alike structure that is also obtained as result of the preprocessing step.  Table 1 shows the comparison of the performance obtained when using seven features and the increased achievement by adding the extra seven.

The article "Pixel-Wise Classification in Hippocampus Histological Images" was published in 2021. Journal: Comput Math Methods Med.

For the remaining seven features, *f*_8_, *f*_9_, ⋯, *f*_14_, the information is extracted from the *I*_NV_ image by following the same process described above, making a total of a 14-D feature vector.

Therefore, one pixel is represented by the 14-D feature space and is denoted by *F*

(11) $$\begin{array}{c} F=\left(f_{1},f_{2},\cdots ,f_{14}\right). \end{array}$$

### 2.3. Data Set Creation

The data set, denoted by *F*_*T*_, is constituted from hippocampal features *F*_*H*_ and nonhippocampal features *F*_*O*_. *F*_*T*_ is distributed in the following way. First, all features *F* from hippocampal pixels are collected from all images, acquiring 24,520 hippocampal features. Then, to be sure to obtain a well-balanced data set, the same amount of randomly picked features is collected from nonhippocampal pixels from all images. Thus, the entire data set *F*_*T*_ makes a total of 49,040 features *F*.

(12) $$\begin{array}{c} F_{T}=F_{H}+F_{O}. \end{array}$$

Next, data set is complemented with ground truth values, *C*_1_ for hippocampal pixel and *C*_0_ for nonhippocampal pixels. For debugging purposes, data set is augmented with *C*_1_ and *C*_0_ pixel coordinates along with the source image name.

Finally, the data set is randomly split into training (*D*_TN_), validation (*D*_VL_), and test (*D*_TS_) set, distributed in 70%, 20%, and 10%, respectively, making sure the same amount of hippocampal features as well as nonhipocampal ones are is contained in these data sets. A sample visual examination conducted on one of the images is shown in Figure 6.

### 2.4. Classification

To be able to determine if a pixel belongs to *C*_1_ or *C*_0_, in this work, different ML models are employed: MLP, RBFN, SVMs, and RF.

A MLP [37] is an artificial neural network that overcomes the limitations of least mean square algorithm in solving prediction problems. MLP consists of a set of three types of nodes: input nodes, known as input layer; one or more layers of computation nodes, known as hidden layer; and an output layer. The first layer receives an input signal and propagates it through network; then, each node of the hidden layer executes a nonlinear activation function, and the result is transmitted to the output layer where nodes located here perform a final activation function whose result is interpreted as the probability that the input signal corresponds to a known class.

The article "Pixel-Wise Classification in Hippocampus Histological Images" was published in 2021. Journal: Comput Math Methods Med.

On the other hand, RBFN was first proposed by Broomhead and Lowe [38] where the hidden layer is trained with an unsupervised algorithm, and the output layer is constructed with a supervised one. The key idea is to transform data points into high-dimensional space with the use of a Gaussian function, so that the transformed points become linearly separable.

SVMs [39] are a category of feed forward networks that can be used for pattern classification and nonlinear regression. SVMs construct a hyperplane as the decision surface in such a way that the margin of separation between positive and negative samples is maximized. There are three main types of SVMs: lineal, polynomials, and radial basis functions.

Random forests [40] are variants of clustering algorithms known as decision trees that perform particularly well on small data sets and like SVMs can perform both classification and regression tasks, but unlike decision trees, RF can limit the sensitivity to small variations in the training data by averaging predictions over many trees.

So that models can be more efficient, techniques such as feature engineering [41] can be used, but looking for maximizing their performance, all *D*_TN_ features, *f*_*i*_ of *F*, are used and standardized making them zero mean and unit variance in the following way.

(13) $$\begin{array}{c} f_{i}=\frac{f_{i}-\mu_{i}}{\sigma_{i}}, \end{array}$$

where *μ*_*i*_ is the average and *σ*_*i*_ is the standard deviation of the *i*-th feature. For all these models, only *f*_*i*_ of *F* features are fed to the models, isolating data that is used for debugging purposes.

In MLP, a supervised learning algorithm known as backpropagation is used for training the layers and the synaptic weight between nodes [37]. With the right choice of weights and with the right number of the hidden nodes, MLP can be used to address classification problems [42]. Hence, the function approximation for classification is defined by a nested set of weighted summations.

RBFN solves the classification problem by proceeding in a hybrid manner. First, an input layer is composed with the same number nodes of the features being evaluated. Then, a hidden layer transforms the given set of nonlinearly separable patterns by applying an unsupervised learning algorithm. Finally, RBFN uses least squares estimation to train the output layer in a supervised manner to solve the classification problem. In RBFN, the function approximation for classification is defined by a single weighted sum [37].

The article "Pixel-Wise Classification in Hippocampus Histological Images" was published in 2021. Journal: Comput Math Methods Med.

RF is settled on decision trees. A decision tree is a machine learning technique, based on the divide and conquer paradigm where the basic idea is to partition the feature space into patches and to fit a model to a patch. RF creates different trees over the same training data set but provides random subset of features to each of the trees in its building process [43] and uses some aggregation technique, such as majority voting to perform the final classification.

SVMs are a type of binary classifiers that construct a hyperplane as the decision boundary and seek to maximize the distance of positive and negative examples given in a training set [37]. SVMs use a two-step process on nonlinearly separable data to find the decision boundary. In the first step, a nonlinear transformation is applied to the data; in the second step, the points that constitute the decision boundary are then determined in the transformed space [44].

There are algorithms used in ML that have been proven to maximize predictive output such as ensemble learning [45]; however, this work is constrained to the mentioned ML models with the purpose of evaluating the pixel characterization method itself.

## 3. Experiments and Results

To measure the algorithmic performance of the proposed method, the before mentioned ML models are trained with *D*_TN_ set, and in order to find the best performing hyperparameters for each model, Random Search and Grid Search techniques are used. The former is used to reduce the search space and the latter to pinpoint the ideal values. Finally, *D*_VL_ set is used to assess that the found hyperparameters produce good results and that models are not overfitted.

The final architecture of the MLP model is implemented with TensorFlow and consists of an input layer with 14 nodes and then four fully connected layers made up with 31, 68, 13, and 7 nodes, respectively, with a ReLU activation type for each one of them. Finally, an output layer consisting of 1 node with a sigmoid activation type constitutes its architecture. The model was compiled using ADAM optimizer and binary cross entropy as loss function (LF) and trained over 37 epochs.

The RBFN is built in TensorFlow with the implementation provided by Vidnerová [46]. It was trained with K-Nearest Neighbourhood (K-NN) for the unsupervised algorithm and backpropagation for the supervised. The model has 3 layers as well. The first layer contains 14 input nodes, the second layer has 71 hidden nodes, and the third layer has one output node with a sigmoid activation type. The same *σ* value is used across Gaussian functions, and it is calculated as follows: $\sigma =d_{\max}/\sqrt{2k}$, where *d*_max_ represents the maximum distance between clusters and *k* is the number clusters, which in turn, match the number of nodes of the second layer. The model used a mean squared error as its LF and RMSprop algorithm for the optimizer and trained over 200 epochs.

The article "Pixel-Wise Classification in Hippocampus Histological Images" was published in 2021. Journal: Comput Math Methods Med.

The rest of the ML models are built with scikit-learn [47]. The best RF model is set with the following hyperparameters: a gini criterion for measuring the quality of splits; a value of $\sqrt{F_{n}}$ is set for the maximum features, where *F*_*n*_ represents the number of features; a value of 1 for the minimum samples per leaf and minimum samples for node split; and unset values for max depth, max leaf nodes, and max samples.

Finally, four different SVM models are used. The first one is configured as lineal support vector classification with these hyperparameters: a value of 182 for the regularization parameter (*C*), a squared hinge LF, and l2 penalty function (PF). The second model is a lineal support vector classification fed with polynomial characteristics, and its hyperparameters are set in the following manner: a value of 172 for *C*, a 2nd degree polynomial characteristic, and a squared hinge LF and a l2 PF. The third model is set with a 3rd degree polynomial kernel; a value of 2.1 for *C*; a squared l2 PF; and a *γ* value of 1/(*C*_*n*_*σ*^2^), where *C*_*n*_ is the number of characteristic and *σ*^2^ is the variance; finally, a value of 40 is used for the independent variable (*b*). The last model uses a radial basis function as kernel type, a squared l2 PF, a value of 1/(*C*_*n*_*σ*^2^) for *γ* parameter, and a value of 182 for *C*.

After finding the best hyperparameter values for each of the models, the *D*_TS_ set is employed to objectively compare the performance of the ML models against each other using the following metrics.

On one hand, the receiver operating characteristic (ROC) curve is used to compare the performance of the classification models by plotting two parameters true positive rate (TPR) and false positive rate (FPR). These metrics are defined by

(14) $$\begin{array}{c} \text{TPR}=\frac{\text{TP}}{\text{TP}+\text{FP}},\\ \text{FPR}=\frac{\text{FP}}{\text{FP}+\text{TN}}, \end{array}$$

where TP means true positives, FN: false negatives, FP: false positives, and TN: true negatives. For this graph, the closer the line is to the upper left corner, the better the classifier is. The ROC curve is displayed in Figure 7.

On the other hand, besides the ROC curve, metrics such as accuracy, precision, recall, and *F*_1_ score are computed with the same purpose. These are defined by

(15) $$\begin{array}{c} \text{Accuracy}=\frac{\text{TP}+\text{TN}}{\text{TP}+\text{TN}+\text{FP}+\text{FN}},\\ \text{Precision}=\text{TPR},\\ \text{Recall}=\frac{\text{TP}}{\text{TP}+\text{FN}},\\ F_{1}\text{score}=2\times \left(\frac{\text{precision}\cdot \text{recall}}{\text{precision}+\text{recall}}\right). \end{array}$$

To evaluate if the added extra seven features resulted in a performance gain, the same data sets *D*_TN_, *D*_VL__,_ and *D*_TS_ are used for all the ML models but are trained, validated, and tested with only the first seven features, respectively.  Table 1 shows that when models use 14 features, all models increase their performance.

The article "Pixel-Wise Classification in Hippocampus Histological Images" was published in 2021. Journal: Comput Math Methods Med.

Table 2 shows all the metrics described before and the values obtained by each model when using 14 features.

In this context, accuracy is a ratio of correctly predicted observation to the total observations; it works better when there is a symmetric data set and if FP and FN have similar cost. When the cost of FP and FN negatives is different, precision and recall metrics need to be considered. The former is the ratio of correctly predicted positive observations to the total predicted positive observations; ergo, it is a good measure to use when the costs of FP are high. The latter, also known as sensitivity, is the ratio of correctly predicted positive observations to all observations in actual class; hence, recall calculates how many of the actual positives the model captures through labelling it as TP. Finally, *F*_1_ score is the weighted average of precision and recall, and it can be selected as the main metric to use when a balance between precision and recall is required and there is an uneven class distribution.

Given that our data set is composed of symmetric quantities between *C*_1_ and *C*_0_ samples and assuming that FP and FN have the same cost, accuracy metric could have picked to evaluate models at one sight. Consequently, the model that presents a better performance is MLP; furthermore, this model also scored the highest on AUC, precision, and *F*_1_ score metrics. However, knowing that all these metrics evaluate models from different perspectives and that the context, in a given problem, plays an important part on deciding which model fits a better solution, the interpretation of the other metrics is important when determining the better model. For this reason, if there was a high cost associated with a FN, i.e., a model predicting that a pixel is *C*_0_ when in fact it is *C*_1_, then recall metric should be the main evaluation metric and for such scenario, RBFN would be the best performing model.

## 4. Discussion

Although good results were obtained with a 7-D and a 5-D feature vectors in the experiments by Marine et al. and Vega et al., respectively, in our experiments, using a 7-D vector did not provide good enough accuracy. This could be, unlike the retinal images that were used in their work, due to the highly variability of the characteristics of the images and the presence of other brain structures that are similar to the seeked hippocampal shape. Nonetheless, when *F* was increased to 14-D, the experiments yielded an average accuracy increase of 2.1285%. This performance increase is associated to the more complete feature set that was generated with our proposed method and the better pixel characterization.

The article "Pixel-Wise Classification in Hippocampus Histological Images" was published in 2021. Journal: Comput Math Methods Med.

The best ML models are described next. For our data set, MLP model achieves the highest value in the accuracy metric and correctly predicts *C*_1_ and *C*_0_ pixels 94.0481% of the time. In contrast, when true positive rate needs to be considered cautiously, only 92.5926% *C*_1_ pixels are correctly predicted and when FN has a greater importance in predicting *C*_1_ pixels, MLP achieves a score of 95.7620%. In this regard, RBFN model achieves the best rate with a 95.9658% value. Finally, for properly predicting *C*_1_ and when an equilibrium between FP and FN is sought, the *F*_1_ score metric is picked. In this regard, the best balance is achieved again by MLP model, with a value of 94.1506%.

Despite that techniques such as deep learning can produce models that achieve higher performance on pixel-wise classification tasks [17, 48], and the architecture for these models tends to be of a much larger size, requiring a vast amount of information and special hardware, as GPUs, to account for the complexity and the computations needed in the training and inference phase execution, in a reasonable amount of time. In this regard, the model studied here already achieves and exceeds the accuracy needed by the subject matter expert to locate the hippocampus and can be probably increased by using ensemble methods [45] and feature engineering techniques [41]. The simplicity of the model means it can do, in a timely manner, fast inferences without the need of special hardware, and for its small size, it can even be implemented in portable devices, such as cell phones or tablets.

Even though this paper is for pixel-wise classification, one could argue that having labelled and located the position of hippocampal pixels, it can be considered as segmentation task. Also, knowing that the work from Mesejo et al. [30] is about hippocampus segmentation and that of Senyukova et al. [32] is for brain structure segmentation, with the hippocampus among them, and that both of them use histological images, we could present a second table to easily compare the results. However, Mesejo et al. use a different definition of accuracy of metric that only takes TP % values; Senyukova et al. present just the result of precision metric without giving further information. For these reasons, a fair comparison table cannot be elaborated but their results are written here for the reader's convenience. Mesejo et al. achieve an accuracy of 92.11% and Senyukova et al. accomplish a precision of 60.7194% for hippocampus structure.

The article "Pixel-Wise Classification in Hippocampus Histological Images" was published in 2021. Journal: Comput Math Methods Med.

## 5. Conclusions

We showed the robustness of the proposed method by evaluating it with different ML models. Furthermore, by adding samples of every image in the data set, we are increasing the exposure to varying styles of histological images. Likewise, by splitting our data set in 70% for training, 20% for validating, and 10% for testing, we can objectively verify that ML models are not overfitting. Hence, we can conclude that the method will be able to generalize when new images are to be presented.

Not only this, the proposed method described in this work showed that it is possible to do pixel-wise classification for histological images and achieve a remarkable good performance too. Furthermore, the described method can significantly reduce the lengthy effort employed by the subject matter expert on identifying and delimiting the hippocampal region and be considered an adequate operation for substituting a manual classification task.

However, there are some aspects that could be considered for future work. One likely way that performance could be improved is by using an ensemble method algorithm. The shown advantage obtained through the use of a 14-D feature vector could be made more efficient by using PCA or a feature engineering technique that reduces the dimensionality of the feature vector and still obtains a good performance. The current method could also be leveraged by fully automating the pixel-wise classification task by integrating an algorithm that locates the hippocampus bounding box. Another direction for future research could be on the generation of a hippocampus segmentation method to further facilitate the measurement of this area and help automating the quantification of hippocampal volume.

## Figures and Tables

**Figure 1:** Coronal sections of the rat brain where the layers of the hippocampus stained with hematoxylin and eosin are observed. 3x magnification. Columns show difference in colour as well as in lighting. Rows show variability in hippocampus shape and markings presence.

**Figure 2:** Diagram of the implemented methodology for hippocampus pixel-wise classification.

**Figure 3:** (a) Original image. (b) Final image: rotated, centred, and resized.

**Figure 4:** (a, d) Colour independence. (b, e) Background homogenization. (c, f) Hippocampus enhancement.

The article "Pixel-Wise Classification in Hippocampus Histological Images" was published in 2021. Journal: Comput Math Methods Med.

**Figure 5:** A hippocampus section is framed with cyan colour. Other brain regions that have a similar shape and similar pixel characteristics are framed with green colour.

**Figure 6:** Red dots represent hippocampus pixels and blue dots represent nonhippocampus pixels. (a) Sample image from training set, (b) the same sample image taken from validation set, and (c) the same sample image taken from test set.

**Figure 7:** ROC curve. Dotted line from bottom left to upper right represents a strictly random classifier.

**Table 1:** Model comparison using 7 vs. 14 features.

Model	Accuracy using 7 features	Accuracy using 14 features	Accuracy difference
MLP	0.917652	0.940481	+0.022829
RBFN	0.915206	0.931512	+0.016306
Random forest	0.915614	0.937627	+0.022013
SVM lineal	0.899715	0.918875	+0.019160
SVM poly feat	0.907868	0.931512	+0.023644
SVM poly kern	0.912556	0.935997	+0.023441
SVM RBF kern	0.917856	0.939462	+0.021606
Total average accuracy	0.912352	0.933638	+0.021285

**Table 2:** Model performance.

Model	Accuracy	AUC	*F*_1_ score	Precision	Recall
MLP	0.940481	0.982761	0.941506	0.925926	0.957620
RBFN	0.931512	0.977904	0.933413	0.908565	0.959658
Random forest	0.937627	0.965623	0.938579	0.924842	0.952730
SVM lineal	0.918875	0.957855	0.920368	0.904088	0.937245
SVM poly feat	0.931512	0.961692	0.932934	0.914319	0.952323
SVM poly kern	0.935997	0.956352	0.937325	0.918623	0.956805
SVM RBF kern	0.939462	0.957067	0.940683	0.922444	0.959658

## Data Availability

Source images, image pixel labels, data set, and code can be found at the following repository: https://github.com/alfonso-vizcaino/hipp_pixel_classification.
